# Colostomy Delays Cell Loss in the Brain and Improves Juvenile Survival in a Neonatal Rat Model of Hirschsprung's Disease

This article has been retracted.

**DOI:** 10.1155/2022/3792798

**Published:** 2022-09-12

**Authors:** Dan Xie, Yitong Du, Yutao Wang, Geoffrey David Hain Croaker, Zheng Zachory Wei, Zan-Min Song

**Affiliations:** ^1^Department of Neurology, Beijing Friendship Hospital Center for Neurological Disorders, Neuroscience Institute, National Clinical Research Center for Digestive Diseases, Beijing, China; ^2^The Eccles Institute of Neuroscience, The John Curtin School of Medical Research and Medical School, Australian National University, Canberra, ACT, Australia; ^3^Department of Clinical Medicine, School of Basic Medical Sciences, Capital Medical University, Beijing, China; ^4^Paediatric Surgery, The Canberra Hospital, Canberra, ACT, Australia

## Abstract

Hirschsprung's disease is a congenital malformation characterized by the absence of enteric ganglia in the distal intestine and gut obstruction. Our previous study indicates the brain pathology during the disease progression. A subpopulation of Hirschsprung's disease patients is also associated with anomalies of the central nervous system. In the investigation, we studied a rat model of Hirschsprung's disease, known as spotting lethal (*sl*/*sl*) ET_B_^−/−^ rats, which carries a spontaneous deletion in endothelin receptor B (human gene name: *EDNRB*) and manifests a similar phenotype as humans with Hirschsprung's disease. Homozygous mutant *sl*/*sl* rats were successfully rescued from premature death by performing colostomy and dramatically survived to their juvenile age. By the body weight measured, their body growth was not revealed to be significantly different between ET_B_^−/−^ and wildtype ET_B_^+/+^ or heterozygous (+/*sl*) ET_B_^+/-^ groups while all underwent the same colostomy. Cell loss was investigated in several brain regions by using terminal deoxynucleotidyl transferase-mediated dUTP nick end-labeling assay (TUNEL) in ET_B_^+/+^, ET_B_^−/−^, and ET_B_^+/-^ rats. Number of TUNEL-positive cells in the cerebellum and the hippocampus of ET_B_^−/−^ rats was significantly increased compared with that of the ET_B_^+/+^ and ET_B_^+/-^ rats. TUNEL-positive cells were observed in the molecular layer and granular cell layers of the cerebellum. In contrast, no significant difference in the density of TUNEL-positive cells was revealed in the cerebral cortex. These results suggest that either endothelin receptor B *sl* mutation or colostomy has predominant lasting effects on the cell survival/loss in the cerebellum and hippocampus of adult ET_B_^−/−^ rats. Our findings provide the information on cellular changes in the brains of patients with Hirschsprung's disease due to congenital *EDNRB* mutation as well as clinically relevant interventions.

## 1. Introduction

The major functions of the intestine are controlled by the enteric nervous system located within the wall of the gut tissue [1]. The absence of enteric neurons can cause a serious medical condition called Hirschsprung's disease [2, 3]. It is a congenital malformation due to a failure of neural crest-derived precursors to colonize intestine during fetal period. The serious consequences include from severe intestinal obstruction to death. Although surgical removal of the blocked intestine saves the lives of Hirschsprung's disease patients, some are complicated with a whole variety of neurological deficits [4]. This indicates that the malformation in Hirschsprung's disease is not limited to the gut but also involves abnormalities in the central nervous system. Our previous reports include a dramatic increase in TUNEL-positive cells in the cerebellum at an early neonatal day 3 of age in rats [5]. The pathological changes are strictly different from neurotropic factor pathways (e.g., BDNF or GDNF). We have previously tested a surgical procedure for prolonging the life of the spotting lethal ET_B_^−/−^ rat [6]. That allows us to further study the long-term neural mechanisms in the developing brain model of Hirschsprung's disease.

The mutation of the gene for endothelin receptor B (human gene name: *EDNRB*) is known to cause both sporadic and familial Hirschsprung's disease in genetically isolated population of Old Order Mennonite [2, 3]. *EDNRB* is the major receptor subtype with the roles in neural cell differentiation, neuronal migration, proliferation, or survival during development [7]. However, little piece of evidence is known about the cellular changes in the brains from Hirschsprung's disease patients. Study of the animal model is useful for the understanding of cellular changes and the potential interventions.

The current study utilizes a strain, known as spotting lethal (*sl*/*sl*) ET_B_^−/−^ rat, which carries a spontaneous deletion of 301 bp within *EDNRB* gene, and manifests a similar phenotype as in humans with Hirschsprung's disease [8, 9]. The ET_B_^−/−^ rats demonstrate a significant decrease in cellular proliferation and an increase in cell death in the cerebellum and the hippocampus/dentate gyrus. *EDNRB*role is critical not only for its effect on the development of the enteric nervous system but also an effect on the development of the brain. Studies on the American MENSA family of Hirschsprung's disease have shown an epilepsy and mental retardation. This phenotype behind an *EDNRB* function remains to be determined [10]. Additionally, due to the genetic lethality of *EDNRB* gene defects, investigation was not focused on the effect of *EDNRB*neural development and the CNS. Our observations based on rat model of enterocutaneous stoma included the effect of *EDNRB* in the developing brain. We curiously tested *EDNRB* deficiency in the rats that led to increased neuronal apoptosis and decreased proliferation in the cerebellum and hippocampus. It was confirmed that *EDNRB* promoted neuronal proliferation and inhibited apoptosis during the development of the nervous system.

However, it was not known whether some of the effects observed in neonatal rats persist into adult life due to inevitable premature death of ET_B_^−/−^ rats. To study the changes in juvenile rats, we performed colostomy on 7-day-old ET_B_^−/−^ rats as previously reported by our group [6]. This surgical operation allowed the contents of the large bowel to be discharged directly through the abdominal wall. The ET_B_^−/−^ rat could live to a juvenile age for our research. In this morphological study, we focused on the effects of *EDNRB* deficiency on cell death in different brain regions of the juvenile ET_B_^−/−^ rat, by comparing with their wild type (+/+) ET_B_^+/+^ or heterozygous (+/*sl*) ET_B_^+/-^ littermates.

## 2. Material and Methods

### 2.1. Experimental Design

Genotyping was done at an earlier age of the rats, for surgical design and grouping during postnatal day 5 (P5) to day 7 (P7). The grouping was randomly performed for colostomy or sham operations after considering genotyping results [8]. The research protocol was modified from our previous article [11], with changes in the surgical conditions considering the study design and the homozygous rats, which usually had poorer nutrition, slower growth, and lighter weight. Compared to the previous protocol, this updated result suggested a much lower mortality rate, consistently showing improved postoperative survival rate. Consequently, it was conducive to any postoperative observation, with extended animal growth to no shorter than postnatal 28 days under surgery. Otherwise, that gene with a fatal mutation was related to the loss of intestine peristaltic function and to the megacolon unable to defecate, leading to water and electrolytes disorder around their P7 to P10 when they barely survived. Our design included colostomy surgeries on the homozygotes to allow the excretion of feces from the stomas throught the abdominal wall. The operated rats survived till skin pigment changes into small black patches and the stomach distention, bowel obstruction and megacolon were relieved.

### 2.2. Animals

Experiments were performed on the Wistar-Imamichi, congenital aganglionosis rat strain that was shown to lack a functional *EDNRB* due to a spontaneous 301 base pair deletion in *EDNRB* gene [9]. Littermates of ET_B_^+/+^, ET_B_^+/-^, and ET_B_^−/−^ rats were generated by heterozygous mating originally from an established colony at the Australian National University animal facilities. The neonatal phenotype for homozygote includes small spotting skin due to reduced cutaneous pigmentation. During P5 to P7, the pups were genotyped as previously performed [8]. All treatment and subsequent operations on rats were approved by the animal ethics committee of the Australian National University.

### 2.3. Colostomy Surgery

Procedures of colostomy in neonatal rats were followed with slight modifications [6]. Briefly, a total of 22 rats of different genotypes at the age of P7 were anesthetized with 2% isoflurane carried in O_2_ at 300 ml/min through an inhalation mask. Abdominal skin was cleaned with chlorhexidine and cetrimide solution (Pfizer Australia) and 70% ethanol. A midline incision was made to minimise faecal soiling and subsequent inflammation of the hind limbs. The proximal colon adjacent to the caecum was pulled through the incision on the abdominal wall. Four sutures along the circumference of the colon wall were anchored to abdominal muscle at the rostral end of incision using absorbable 8-0 braided coated Vicryl (Ethicon Inc.). At about 0.5 cm distal to this sutured region, another segment was similarly sutured to the caudal end of the incision. The bowel was severed in between to perform two colostomies. Both were further fixed to the skin using the 6-0 nonabsorbable polypropylene monofilament suture (Ethicon Inc.). The skin between the two colostomies was closed using 6-0 suture. Wound was applied with Wound-Gard (Virbac Pty Ltd., Australia), a bitter tasting antiseptic cream, to prevent the mother from licking the wound and cannibalism, which occurred for eight rats without the cream application. After regaining consciousness, the pups were wiped thoroughly with the mother's bedding and faecal pellets before being returned to the mother, together with unoperated pups in the same cage. Postoperated rats were then monitored on a daily basis. Warm saline-soaked cotton tips were used to remove dried faecal matter blocking the stoma. All operated pups were weaned at P21 after birth and fed with normal rat chow for additionally one week. Body weights were recorded at P28 and brain tissue was collected according to our previous study [11]. We were able to collect data from fourteen rats with colostomy (four ET_B_^+/+^ rats, six ET_B_^+/-^ rats, and four ET_B_^−/−^ rats).

Sham operations were performed in additional five ET_B_^+/+^ rats, which entailed incising abdominal wall, followed by gently handling the intestine and suturing the wounds. Those rats were handled in the same way with the others receiving the colostomy. With our surgical interventions, the survival rate of the animals detected at P28 was around 66.7%.

### 2.4. Tissue Preparation and TUNEL Assay

The effect of *EDNRB* deficiency on cell death in the juvenile rat brain was assessed using terminal deoxynucleotidyl transferase-mediated dUTP nick end-labeling (TUNEL). Four to six rats for each genotype and operations (ET_B_^+/+^ with colostomy, ET_B_^+/-^ with colostomy, and ET_B_^−/−^ with colostomy) were examined at the age of P28 (three weeks after colostomy). Rats were sacrificed after i.p. injection of pentobarbital at 100 mg/kg and transcardial perfusion-fixed with 4% paraformaldehyde. Brains were dissected and postfixed and coronal sections were made at 12 *μ*m on a cryostat. Three to four random sections from each region of the rat were processed for TUNEL with recombinant terminal transferase (Roche Diagnostics, Cat. 03333574001) combined with biotinylated dUTP (Roche, Cat. 11093070910), followed with streptavidin conjugated Alexa Fluor 594 (Invitrogen, Cat. S32356). Sections were counterstained with DAPI (300 nM in PBS).

### 2.5. Image Analysis

Fluorescence images of TUNEL-stained sections were examined under Nikon A1 confocal microscope system with appropriate filter sets. Images were collected from three to four random sections in each region for cell counting using ImageJ (1.46r; W. Rasband, NIH, USA) within the cerebellum, the hippocampus/dentate gyrus, and the cerebral cortex. All cell counting was carried out by experimenters blinded to the genotype.

### 2.6. Cell Culture and Western Blot Analysis

Human SH-SY5Y cell line was applied to confirm the roles of the *EDNRB* mutations in the neural-like cells. The culture conditions were used according to protocols with slight modification [12]. Cells were maintained in RPMI-1640 medium (Life Technologies, USA), supplemented with 10% fetal bovine serum (Hyclone, USA) and 100 U/ml penicillin/streptomycin (ABAM Life Technologies, California, USA) at 5% CO_2_, 37°C with humidified air in an incubator. Transfection was performed and plasmid provided by Dr. Jinling Huang (Peking University; Hechuang Biotech, Guangzhou, China) with human cell line *EDNRB* gene nucleotide deletion of GTGCCTAAAGGAGACAGGACGGCAGGATCTCCGCCACGCACCATCTCCCCTCCCCCGTGCCAAGGACCCATCGAGATCAAGGAGACTTTCAAATACATCAACACGGTTGTGTCCTGCCTTGTGTTCGTGCTGGGGATCATCGGGAACTCCACACTTCTGAGAATTATCTACAAGAACAAGTGCATGCGAAACGGTCCCAATATCTTGATCGCCAGCTTGGCTCTGGGAGACCTGCTGCACATCGTCATTGACATCCCTATCAATGTCTACAAG according to matching of the rat gene nucleotide sequence reported [9]. The *EDNRB* gene was mutated via the transfection using Lipofectamine 3000 kit. After medium change, the cells were then supplemented with 100 *μ*g/ml G418 (Life Technologies).

The protein sample was collected from control cell lines or *EDNRB* mutation cell lines. We performed the experiments according to our previous publication with minor modifications [13]. The cells were scratched and lysed on ice in RIPA buffer (20 mM pH 7.5 Tris-HCl, 150 mM NaCl, 1 mM Na_2_EDTA, 1 mM EGTA, 1% Triton, 2.5 mM sodium pyrophosphate, 1 mM beta-glycerophosphate, 1 mM Na_3_VO_4_, 1 *μ*g/ml leupeptin, and 1 mM phenylmethylsulfonyl fluoride). With 30 min incubation in EP tubes, the cell lysates were centrifuged at 12,000 × *g* for 30 min at 4°C. Supernatant was then collected. Protein concentration in the solution was determined using a Coomassie Brilliant Blue protein assay kit (Bio-Rad). Western blot was carried out and AEP antibody 6E3 as previously described [14].

### 2.7. Statistical Analysis

Results of body weight and number of dead cells (e.g., TUNEL-positive cells per mm^2^) were presented as the mean ± SEM. For statistical analysis of data from different genotypes, one-way analysis of variance (ANOVA) was used followed by a Tukey's multiple comparison test (Prism 5, GraphPad, CA, USA) unless otherwise specified. Differences were considered significant at *P* < 0.05.

## 3. Results

### 3.1. The Effect of Colostomy on the Body Growth of Rats

Our previous study showed that colostomy was able to rescue ET_B_^−/−^ rats that would otherwise die early due to gut blockage and subsequent malnutrition [6]. We performed colostomy surgery on the P7 rats (Figure 1). The weight gain of four groups of rats was compared at 28 days old (three weeks after colostomy). In rats that received colostomy, the averaged body weight in ET_B_^−/−^ rats was lower than that in ET_B_^+/+^ rats or ET_B_^+/-^ rats, although it did not reach a statistically significant level (Figure 2). However, colostomy operation per se did affect body weight, since the weight of ET_B_^+/+^ group with sham operations was significantly higher than ET_B_^+/+^ rats with colostomy. The human cell culture experiments further suggested that there were not dependent on either BDNF or GDNF (*P* > 0.05, Figure S1) in the cells with mutated *EDNRB*, consistent with our previous reports in the animal model. We assumed that colostomy operation compromised body growth, probably due to decreased fluid and electrolyte absorption and accelerated gastric emptying but showed protection of the brain.

### 3.2. Significant Cell Loss in the Cerebellum in ET_B_^−/−^ Rats

To evaluate the detrimental cell death effect of the mutated *EDNRB*, TUNEL-positive nuclei were stained and compared among four groups of juvenile rats: ET_B_^+/+^ with colostomy, ET_B_^+/-^ with colostomy, and ET_B_^−/−^ with colostomy under genotyping (Figure S2). The Purkinje cell nuclei with DAPI labeling were located between the molecular layer and the granular cell layer. TUNEL-positive nuclei were found in the cerebellum of ET_B_^+/+^ rats (Figures 3(a)–3(f)). Significantly higher number of TUNEL-positive nuclei per section was revealed in the same region of ET_B_^−/−^ rats with colostomy (Figures 3(e) and 3(f)).

By examining the four layers of the juvenile cerebellum (Figure 3), the largest proportion of TUNEL-positive cells in ET_B_^−/−^ rats were located in the molecular layer, followed by the granular cell layer. The white matter and Purkinje cell layer had occasional TUNEL-positive cells. It might be interesting to notice that the proportion remained similar across different genotypes and no statistically significant difference was found in any layers between each of the four genotypes (data not shown). Those results indicated that *EDNRB* mutation could be consistently/broadly involved in apoptosis in the cerebellum of juvenile ET_B_^−/−^ rats.

### 3.3. Significant Cell Loss in the Hippocampus/Dentate Gyrus in ET_B_^−/−^ Rats

The cerebral cortex, the dentate gyrus, and the hippocampus were examined among normal, ET_B_^+/-^ and ET_B_^−/−^ genotypes littermates. TUNEL-positive nuclei were found in CA1 to CA3 regions of the hippocampus and the dentate gyrus of ET_B_^+/+^ rats (Figure S3). In contrast, density of TUNEL-positive nuclei in the hippocampus/dentate gyrus was significantly higher in ET_B_^−/−^ rats than in ET_B_^+/+^ rats with colostomy. Little difference in the hippocampus was seen between ET_B_^+/+^ and ET_B_^+/-^ or between ET_B_^+/-^ and ET_B_^−/−^ groups of juvenile rats. Interestingly, pursuing our previous design, there was no increased level of BDNF or GDNF (data not shown), two growth factors that contribute to brain development and repair greatly.

### 3.4. Cell Loss in the Cerebral Cortex

Few TUNEL-positive cells were found in the cerebral cortex of juvenile rats (Figure 3(g)). There was no significant change between each of the groups and ET_B_^−/−^ animals received colostomy. These results indicated that the loss of functional *EDNRB* had little relation with the cell death in the cerebral cortex of juvenile rats. Consistently, the animal survival was dramatically improved (Figure 4).

## 4. Discussion

In Hirschsprung's disease (or congenital aganglionic megacolon), it occurs with abnormal development of intestinal neurons (ganglion cells) and delayed progression of stool through the intestines. Following surgical procedures in clinic, it is commonly observed for children with Hirschsprung's disease to have few problems [15]. Based on evidences from abdominal x-ray, contrast enema, and rectal biopsy, the pathological gut segment can be removed by the surgery. There are usually few follow-up interventions although neurodevelopmental issues of the children are documented [16]. The clinical follow-up studies have limitations. Understanding the disease progression in central nervous system research is useful for the further exploration of neurodevelopment mechanisms and treatment [17].

Our previous collaborational study has shown that ET_B_^−/−^ rats can be rescued from premature death when colostomy is performed at the neonatal period [6]. This operation enables us to keep ET_B_^−/−^ rats survive up to four to six weeks when they are sacrificed. The present study confirms that ET_B_^−/−^ rats (which would otherwise die) have similar weight gain as their ET_B_^+/+^ and ET_B_^+/-^ littermates that receive the same colostomy surgery. This indicates that the effects on cell death in the brain are unlikely related to malnutrition. However, rats with colostomy have significantly lower body weight than sham-operated ET_B_^+/+^ rats, which suggests that colostomy per se compromises body growth. The mechanisms are related to decreased fluid and electrolyte absorption and accelerate gastric emptying as in human with colostomy. Therefore, the comparison of brain development has to be between different genotypes with colostomy. There was no difference in behaviors as well as the general body size of the rats.

The effect of null mutation of *EDNRB* was further examined for cell death in the cerebellum, the cerebral cortex, the dentate gyrus, and the hippocampus by comparing ET_B_^−/−^, ET_B_^+/-^, and ET_B_^+/+^ littermates that received colostomy. The deficiency of *EDNRB* substantially increased cell death in the cerebellum, hippocampus, and dentate gyrus of juvenile ET_B_^−/−^ rats, compared with ET_B_^+/+^ littermates. However, no such change was observed in the cerebral cortex.

*EDNRB* receptor expression is differentially regulated during early and later brain development. In embryos, *EDNRB* is abundantly expressed in cells lining the ventricles, but its expression is substantially decreased in the cortex and subventricular zones at P14 [18]. In contrast, the expression of *EDNRB* in the cerebellum and hippocampus persists in juvenile rats [19]. *EDNRB* is generally related to the development of neural crest lineage. Growing evidence shows its regulatory effects on a number of regions of the brain, including the cerebellum, hippocampus, and early cerebral cortex. This study further shows pathological cell death persisting in juvenile ET_B_^−/−^ rat cerebellum and hippocampus where *EDNRB* is normally expressed at this age [20]. We have not observed a significant increase in cell death of the cerebral cortex, which is consistent with significant decrease in the *EDNRB* expression within the first two weeks following birth [21]. Taken together, the mutated *EDNRB* effects in different regions of the brain further support a receptor mediated event during development. Variants have been identified in the RET/EDNRB pathways, accounting for 30% of any sporadic Hirschsprung's disease cases [22]. Unfortunately, our study may not provide direct targets for clinical applications. The signaling pathways are followed and the research will be reported in our further paper.

Hirschsprung's disease is associated with a variety of congenital abnormalities in the CNS, including microcephaly, agenesis of the corpus callosum, asymmetry of lateral ventricles, central hypoventilation, sensorineural deafness, seizures, mental retardation, and autonomic nervous abnormalities [23–25]. Although Hirschsprung's disease in humans is polygenic, the *EDNRB* mutation causes a substantial proportion of sporadic and familial cases [26–28]. The currently reported brain structural changes have not been studied in human brains with Hirschsprung's disease. Our results in ET_B_^−/−^ rats may allow us to extrapolate that the major effects on human Hirschsprung's disease with congenital *EDNRB* mutation are associated with early development and an increased cell death within the cerebellum and the hippocampus. In addition, cerebral cortical cell protection may be critically important to the juvenile survival in the disease, which are explored further by our group.

## 5. Conclusion

The *sl*/*sl* ET_B_^−/−^ rats were rescued from premature death by performing colostomy. Cell loss significantly occurred in the cerebellum and hippocampal formation of juvenile ET_B_^−/−^ rats. ENDRB mutation could possess long lasting effects on the cell death in the cerebellum and hippocampus. Our findings would help improve the understanding of cellular changes in the brains of Hirschsprung's disease patients with congenital *EDNRB* mutation as well as clinically relevant interventions.

## Figures and Tables

**Figure 1:** The surgery procedure and experimental design. P0/5/7/28: postnatal day 0/5/7/28.

**Figure 2:** Body weight after colostomy surgery. Comparison of the body weight of ET_B_^+/+^ rats without colostomy (sham operated) and ET_B_^+/+^ rats, ET_B_^+/-^ rats, or ET_B_^−/−^ rats with colostomy. The colostomy surgeries were performed at P7 and the body weights were measured at an age of 28 days. All rats with colostomy had comparable body weights regardless of their genotypes. We observed a slight lighter in all the operated rats than the ET_B_^+/+^ rats without colostomy. Importantly, colostomy saved ET_B_^−/−^ rats till at least 28 days after birth, compared to a barely survival rate among ET_B_^−/−^ rats without colostomy (data not shown).

**Figure 3:** Cell death analysis in the brain regions. Representative confocal images of transverse sections of the cerebellum of the juvenile rats indicated the brain regions showing TUNEL-positive nuclei (red) with DAPI counterstaining (blue). The structure of juvenile cerebellum was revealed with DAPI staining, where molecular layer, granular cell layer, and white matter were clearly recognizable. (a) Lower magnification view of a section from sham-operated ET_B_^+/+^ rat showing folia. (b) Higher magnification view of the same section showing the molecular layer, granular cell layer, white matter, and Purkinje cell layer. (c and d) Occasional TUNEL-positive nuclei are found in granular cell layer and the molecular layer in ET_B_^+/+^ rats and in ET_B_^+/-^ rats with colostomy. (e) Substantially higher density of TUNEL-positive nuclei were located in the molecular layer of the ET_B_^−/−^ rats but very few in granular and Purkinje cell layers. Scale bar, 200 *μ*m (a) and 20 *μ*m (b–e). Summary data on the density of TUNEL-positive nuclei in the cerebellum (f) and cerebral cortex (g) of rats from different genotypes. Averages from 4-6 rats in each genotype were compared with one-way ANOVA, specifically Kruskal-Wallis test with Dunn's multiple comparisons test (for (g)), where ∗ denotes *P* < 0.01.

**Figure 4:** Survival rates after colostomy surgery.

## Data Availability

The datasets used and/or analysed during the current study are available from the corresponding author on reasonable request. The morphological and biochemical data used to support the findings of this study were supplied by D.X. and Z.S. under license and so cannot be made freely available. Requests for access to these data should be made to Z.S. at z.song@griffith.edu.au.

## Additional Points

*Highlights*. (i) Colostomy rescued rats with Hirschsprung's disease (spotting lethal rats) from premature death. (ii) Cell loss significantly occurred in the cerebellar and hippocampal regions of juvenile spotting lethal rats. (iii) Colostomy with endothelin receptor B *sl* mutation in the rat could be associated with protection of cerebral cortical cells.

## Supplementary Materials

Supplementary 1 Figure S1: protein level analysis of human cell line with *EDNRB* deletion mutation. The relative protein levels were compared based on the protein samples of human SH-SY5Y cell lyses. The *EDNRB mut* experiments indicated the deletion mutation in the cells, in which *EDNRB* protein expression was detected significantly low (A). Neither BDNF (B) nor GDNF (C) was changed.

Supplementary 2 Figure S2: representative images showing related phenotype of the ET_B_^−/−^ rat. In the rats with congenital *EDNRB* gene defects, we recorded the consequences due to the intestinal obstruction with malnutrition and electrolyte disorders, or peritoneal infections. Mostly, the neonatal rats with homozygous mutations could die within one week of birth. We first applied colostomies to the *EDNRB* gene defective neonatal rats after genetic testing of the newborn ones. It was allowed to observe the cellular apoptosis and proliferation as well as the animal survival of ET_B_^−/−^ rats for the body growth and nervous system development. With the surgical interventions, ET_B_^−/−^ neonatal rats survived to adulthood. Importantly, with/without the operation on the rats with congenital *EDNRB* gene defects, there were both changes in hair melanin pigmentation (A and B). Typically, there were 200 bp and 500 bp gene fragments for ET_B_^+/-^, the  bp alone for ET_B_^+/+^, and the 500 bp alone for ET_B_^−/−^ rats (as shown in C).

Supplementary 3 Figure S3: representative images of the hippocampus of a juvenile ET_B_^−/−^ rat with colostomy showing the distribution of TUNEL-positive nuclei (red) with DAPI counterstaining. (A–C) Low magnification view of the hippocampus (including CA1 and CA3) and dentate gyrus. (D-I) TUNEL-positive nuclei were visible in all the three brain regions of ET_B_^−/−^ rats. Scale bar: 50 *μ*m for (C) and 20 *μ*m for (F) and (I). (J) Summary data comparing the density of TUNEL-positive nuclei in the hippocampus of juvenile ET_B_^+/+^, ET_B_^+/-^, and ET_B_^−/−^ rats. ET_B_^−/−^ rats had significantly more TUNEL-positive cells than ET_B_^+/+^ rats (^∗^*P* < 0.05). However, no significant difference in the cerebral cortex was found between any groups of the rats (*P* > 0.05).
